# Mineral Composition, Phenolic Content, and *In Vitro* Antidiabetic and Antioxidant Properties of Aqueous and Organic Extracts of *Haloxylon scoparium* Aerial Parts

**DOI:** 10.1155/2021/9011168

**Published:** 2021-10-14

**Authors:** Nacima Lachkar, Fatima Lamchouri, Khadija Bouabid, Mohamed Boulfia, Souad Senhaji, Mourad Stitou, Hamid Toufik

**Affiliations:** Laboratory of Natural Substances, Pharmacology, Environment, Modeling, Health & Quality of Life (SNAMOPEQ), Polydisciplinary Faculty of Taza, Sidi Mohamed Ben Abdellah University of Fez, B.P.: 1223 Taza-Gare, Taza, Morocco

## Abstract

*Haloxylon scoparium* is a plant widely used in traditional medicine for the treatment of diabetes. Hence, this study focuses on the mineralogical and chemical composition and evaluation of the antidiabetic and antioxidant activities of the aerial part of this species. The mineralogical analysis was done by inductively coupled plasma atomic emission spectrometry (ICP-AES). The phytochemical study consisted in the preparation of different extracts from the aerial part by aqueous and organic extraction using Soxhlet and cold maceration. Then, phytochemical screening was performed on the plant powder and on the extracts, which is completed by spectrophotometric quantification of total polyphenols, flavonoids, and catechic tannins. The evaluation of antidiabetic activity was done by three enzymes: *a*-amylase, *a*-glucosidase, and *ß*-galactosidase, and that of antioxidant activity was done by five methods: H_2_O_2_, DPPH, ABTS, FRAP, and reducing power (RP). Mineralogical analysis revealed the presence of iron, potassium, magnesium, phosphorus, sodium, copper, calcium, strontium, selenium, and zinc. The studied part is rich in alkaloids, flavonoids, catechic tannins, and saponins. The methanolic extract is rich in total polyphenols (161.65 ± 1.52 Ug EAG/mg E), and the ethyl acetate extract has high levels of catechic tannins (23.69 ± 0.6 Ug EC/mg E). In addition, the decoctate expresses a high flavonoid content of 306.59 ± 4.35 Ug EQ/mg E. The *in vitro* evaluation of the antidiabetic activity showed that the decoctate has a higher inhibitory capacity on *a*-glucosidase (IC50 = 181.7 ± 21.15 ug/mL) than acarbose (IC50 = 195 ± 6.12 ug/mL). The results of the antioxidant activity showed that the methanolic extract and the decoctate present a percentage of hydrogen peroxide (H_2_O_2_) scavenging (20.91 ± 0.27 and 16.21 ± 0.39%) higher than that of ascorbic acid (14.35 ± 0.002%). Positive correlations obtained between the total polyphenol content and the antioxidant activity of the extracts were studied. A positive correlation of *a*-amylase inhibitory activity was also recorded with the antioxidant activity tests.

## 1. Introduction

Oxidative stress causes adverse effects on human health and can be the cause of several diseases such as cancer, diabetes, and cardiovascular diseases [1]. It is also responsible for respiratory distress syndrome [2].

Antioxidants are able to combat this oxidative stress and prevent free radical damage, and antioxidant-rich micronutrients can help prevent cancer and diabetes [3]. Some minerals are involved in the regulation of insulin secretion and the insulin signalling pathway influencing insulin sensitivity [4]. Antioxidant molecules in plants protect against complications of type 2 diabetes [5] and protect against cardiovascular disease, atherosclerosis, and hypertension [6].

Among the sources of antidiabetic and antioxidant molecules available in nature, there are medicinal plants that are frequently used in traditional herbal medicine, which are reputed to be effective in treating several diseases. Hence, it is important to expand research on natural antioxidants of plant origin.

*Haloxylon scoparium* is a medicinal plant that belongs to the Chenopodiaceae family, which has 120 genera and more than 1300 species [7], and is a small, highly branched shrub distributed in North Africa, southeastern Spain, and parts of Iran, Turkey, Iraq, and Syria [8]. Several ethnobotanical and ethnopharmacological surveys have shown that *Haloxylon scoparium* is used in Moroccan traditional medicine against several diseases such as hypertension and diabetes [9,10]. Previous work in our laboratory has shown that *H. scoparium* does not have antifungal activity, and of different organic extracts tested (methanol, chloroform, ethyl acetate, and petroleum ether), only the ethyl acetate extract has moderate antibacterial activity (7–12 mm) against the *Staphylococcus aureus* strain [7].

In the present study, we were interested in the mineralogical investigation by determining the mineral content of the aerial part of *Haloxylon scoparium*, phytochemical investigation by preparing different aqueous (decocted, infused, and macerated) and organic extracts using solvents of decreasing polarity (methanol, chloroform, ethyl acetate, and petroleum ether), the characterisation of the composition of secondary metabolites by carrying out a phytochemical screening on both the powder and the different aqueous and organic extracts prepared, and finally the quantification of phenolic compounds contained in the aerial part of *Haloxylon scoparium*. The biological and pharmacological study consisted of an *in vitro* evaluation of the antidiabetic activity of the prepared aqueous and organic extracts by the three enzyme inhibition tests of *a*-amylase, *a*-glucosidase, and *ß*-galactosidase, and that of the antioxidant capacity using five tests: hydrogen peroxide (H_2_O_2_) scavenging test; DPPH (2,2-diphenyl-1-picrylhydrazyl) free radical scavenging test; ABTS (2,2-azinobis (3-ethyl-benzothiazoline-6-sulphonate) or TEAC (Trolox equivalent antioxidant capacity) test; iron reduction antioxidant power (FRAP) test, and the reducing power (RP) test. To investigate the correlations between the chemical composition of the different extracts and the antioxidant and antidiabetic activities, we used principal component analysis (PCA).

## 2. Materials and Methods

### 2.1. Plant Material

The plant material consists of the aerial part of *Haloxylon scoparium* collected in July 2019 near the region of Taddart located 42.1 km from the city of Taza (geographical coordinates: N 34°12.530′, W 003°32.917') (Figure 1).

The botanical identification of the plant *Haloxylon scoparium* was carried out by Dr. Abdelmajid Khabbach at the Laboratory of Natural Substances, Pharmacology, Environment, Modeling, Health and Quality of Life (SNAMOPEQ), Polydisciplinary Faculty of Taza (FPT), Sidi Mohamed Ben Abdellah University of Fez (USMBA), B.P.: 1223, Taza-Gare, Taza, Morocco. A reference sample (ST2019/07) of the plant was deposited in the herbarium of the SNAMOPEQ laboratory of the FPT.

### 2.2. Mineralogical Study

Quantitative mineralogical analysis was carried out by inductively coupled plasma atomic emission spectroscopy (ICP-AES), which is a multielement analytical method that allows the measurement of several elements while using the quantitative measurement of the optical emission from the stimulated atoms, to determine the concentration of the analyte. It was carried out according to the protocol of Arora et al. [11], where 0.5 g of the powder of the aerial part of *Haloxylon scoparium* was placed in test tubes, a solution of perchloric acid and nitric acid (1 : 4) was added to digest the mixture, and then the samples were placed in the oven at 80°C. The samples were then allowed to cool, and the contents were filtered through Whatman filter paper. The sample solution was made up to a final volume of 25 ml with distilled water and analysed by HORIBA Jobin Yvon inductively coupled plasma atomic emission spectrometry (ICP-AES) [11].

### 2.3. Phytochemical Study

#### 2.3.1. Preparation of Aqueous and Organic Extracts

The bioactive content of the aerial part of *Haloxylon scoparium* was extracted by two processes: an aqueous extraction using distilled water according to 3 modalities: decoction, infusion, and maceration, and another organic one in hot Soxhlet using organic solvents of different polarities: methanol, chloroform, ethyl acetate, and petroleum ether and in cold by maceration with methanol. The extraction methodology used is described in our previous work [12–16]. After removal of the solvents using a rotary evaporator (Buchi R-210), extraction yields were calculated and all extracts obtained were weighed and stored at 4°C.

#### 2.3.2. Phytochemical Screening

The families of secondary metabolites such as catechic tannins, gall tannins, flavonoids, saponins, alkaloids, anthracenosides, free quinones, and anthraquinones were searched in the powder of the plant material and in the aqueous and organic extracts prepared from the aerial part of *Haloxylon scoparium* by staining and precipitation reactions as described in previous works of our laboratory [12–16].

#### 2.3.3. Determination of Phenolic Compounds

The quantitative analysis was based on the results obtained by phytochemical screening; the determination of total polyphenols, flavonoids, and catechic tannins was carried out on the aqueous and organic extracts of the aerial part of *Haloxylon scoparium* as defined in previous publications of our laboratory [12,14–16].

#### 2.3.4. Determination of Total Polyphenols

The determination of total polyphenols in extracts from the aerial part of *Haloxylon scoparium* was carried out according to the Folin–Ciocalteu reagent method [17] as presented in our previous articles [13–16].

#### 2.3.5. Determination of Flavonoids

Total flavonoids were quantified using the method adapted by Mihai et al. [18] using aluminium trichloride and sodium hydroxide; the protocol is referred to in previous works [13–16].

#### 2.3.6. Determination of Catechic Tannins

Catechic tannins are determined by the vanillin method based on the ability of vanillin to react with condensed tannins in the presence of acid to form a coloured complex measurable at 500 nm. The procedure has been described previously in [13–16,19].

### 2.4. *In Vitro* Study of Antidiabetic Activity

#### 2.4.1. Inhibitory Activity of the Enzyme *a*-Amylase

The *a*-amylase inhibitory power of our aqueous and organic extracts was found *in vitro* by colorimetric assay based on the quantification of glucose released into the reaction medium. Because of the reducing properties of sugar, 3,5-dinitrosalicylic acid which acts as an oxidant is reduced to 3-amino-5-nitrosalicylic acid [20]. A mixture of 200 *μ*L of sample and 200 *μ*L of 0.02 M sodium phosphate buffer (pH = 6.9) containing the enzyme *a*-amylase (10 U/mL) was incubated at 30°C for 10 min. Then, 200 *μ*L of 1% starch solution was added to the reaction mixture. The mixture was incubated at 30°C for 3 min. Then, 1 mL of the solution (DNS) was added and the reaction mixture was incubated at 90°C for 10 min. The reaction mixture was then diluted by adding 5 mL of distilled water, and the absorbance was measured at 540 nm in the type spectrophotometer (UviLine 9100–94000 UV/Vis). Acarbose was used as a positive control.

#### 2.4.2. Inhibitory Activity of the Enzyme *a*-Glucosidase

The effect of our aqueous and organic extracts on the catalytic activity of *a*-glucosidase was identified according to the method in [21]. A mixture of 150 *μ*L of the sample and 100 *μ*L of 0.1 M sodium phosphate buffer (pH = 6.7) containing the *a*-glucosidase enzyme solution (0.1 U/mL) was incubated at 37°C for 10 min. After preincubation, 200 *μ*L of 1 mM pNPG solution in 0.1 M sodium phosphate buffer was added. The reaction mixtures were incubated at 37°C for 30 min. After incubation, 1 mL Na_2_CO_3_ (0.1 M) was added and we measured the absorbance at 405 nm using the spectrophotometer (UviLine 9100–94000 UV/Vis). The inhibitory activity of *a*-glucosidase was expressed as percentage inhibition, and IC50 values were determined. Acarbose was used as a positive control.

#### 2.4.3. Inhibitory Activity of the Enzyme *ß*-Galactosidase

The *in vitro ß*-galactosidase inhibition assay was done by colorimetric assay [22]; for this, a volume of 150 *μ*L of different extracts and 100 *μ*L of sodium phosphate buffer (0.1 M) at pH = 7.6 containing *ß*-galactosidase enzyme solution (1 U/mL) was incubated at 37°C for 10 min. Afterwards, we added 200 *μ*L of the substrate 2-nitrophenyl beta-D-galactopyranoside (1 mM) prepared in sodium phosphate buffer (0.1 M) at pH = 7.6. The mixtures were incubated at 37°C for 30 min. After incubation, we added 1 mL Na_2_CO_3_ to stop the reaction and recorded the absorbance at 410 nm using a spectrophotometer. Quercetin is used as a positive control.

The results of the three tests for antidiabetic activity were expressed as %inhibition and calculated using the following equation:

(1) $$\begin{array}{c} \text{\% inhibition}=\left(\frac{\left(\left(\text{Ac}\left(+\right)-\text{Acb}\left(-\right)\right)-\left(\text{As}-\text{Ab}\right)\right)}{\left(\text{Ac}\left(+\right)-\text{Acb}\left(-\right)\right)}\right)*100\text{,} \end{array}$$

where Ac**+** is the absorbance of control with enzyme, Ac- is the absorbance of control without enzyme, As is the absorbance of sample with enzyme, and Ab is the absorbance of sample without enzyme

### 2.5. *In Vitro* Study of Antioxidant Activity

Five methods were chosen to evaluate the antioxidant activity of the aqueous and organic extracts of the aerial part of *Haloxylon scoparium*, namely, hydrogen peroxide (H_2_O_2_) scavenging test, DPPH (2,2-diphenyl-1-picrylhydrazyl) free radical scavenging test, ABTS (2,2-azinobis (3-ethyl-benzothiazoline-6-sulphonate) or TEAC (Trolox equivalent antioxidant capacity) test, iron reduction antioxidant power (FRAP) test, and the reducing power (RP) test.

#### 2.5.1. Hydrogen Peroxide (H_2_O_2_) Scavenging Activity

The evaluation of H_2_O_2_ scavenging capacity was carried out by the method described by Ruch and coworkers [23]: The experimental protocol has been detailed by previous works [13–16]. The percentage of hydrogen peroxide scavenging was determined by the following formula:

(2) $$\begin{array}{c} \text{\%}=\left[\frac{\left(\text{AC}-\text{AE}\right)}{\text{AC}}\right]\times 100\text{,} \end{array}$$

where AC is the absorbance of the control and AE is the absorbance of the sample.

#### 2.5.2. DPPH Free Radical Scavenging Test

The test for the scavenging of the DPPH radical (2,2-diphenyl-1-picrylhydrazyl (C18H12N5O6)) radical from the aerial part of *Haloxylon scoparium* was performed according to the protocol described by previous works [13–16,24]. The results obtained are compared with Trolox, BHT, and ascorbic acid which are employed as standard antioxidants. For each extract, the test is repeated three times.

The results are expressed as percentage inhibition using the following formula:

(3) $$\begin{array}{c} I\left(\text{\%}\right)=\left[\frac{\left(\text{Abs}-\text{Abss}\right)}{\text{Abs}}\right]\times 100\text{,} \end{array}$$

where *I*(%) denotes the percentage inhibition, Abs is the absorbance of the negative control, and Abss is the absorbance of the sample.

The percentage of inhibition allowed us to establish a linear regression curve linking the different concentrations and the percentages of inhibition, and from this curve, we determined the IC50, the concentration that results in 50% inhibition of the DPPH• radical.

#### 2.5.3. Equivalent Antioxidant Capacity of Trolox (TEAC or ABTS)

The inhibitory power of the ABTS^•+^ radical is evaluated by the method described by Re et al. in 1999 [25]. For detailed protocol, refer to our previous works [13–16]. The reading is taken at 734 nm by using a spectrophotometer (UviLine 9100–94000 UV/Vis). Trolox is used as a standard, and the results obtained are expressed as mg Trolox equivalent per gram of extract (mg TE.g-1E).

#### 2.5.4. Ferric Reducing Antioxidant Power (FRAP) Assay

The antioxidant capacity of the tested extracts was determined based on the method of Benzie and Strain [26]. The experimental protocol was detailed in our previous work [13–16]. The antioxidant capacity of the different extracts is represented as mg Trolox equivalent/g extract (mg TE.g-1E).

#### 2.5.5. Reducing Power Assay

The reducing power of our extracts was determined according to the method described by [13–16,27], based on the reduction of ferric iron Fe^3+^ to ferrous iron Fe^2+^. The absorbance reading was taken at 700 nm. Ascorbic acid was used as a positive control. The final result is represented as milligrams of ascorbic acid equivalent per gram of extract.

### 2.6. Statistical Analysis and Principal Component Analysis (PCA)

The statistical study was carried out using the statistical software GraphPad Prism 5. All experiments were performed in triplicate. The results are expressed as mean ± SEM. The results are analysed by the one-way ANOVA test followed by the Tukey test for multiple comparisons and determination of significance levels. Values of *p* ≤ 0.05 are considered statistically significant.

Principal component analysis (PCA) was used to analyse the relationships between the chemical composition of the aqueous and organic extracts tested and the biological activities and also to better visualise the correlations between the chemical composition of the eight prepared *Haloxylon scoparium* extracts and their antidiabetic and antioxidant activity *in vitro*.

## 3. Results

### 3.1. Mineralogical Study of the Aerial Part of *Haloxylon scoparium*

The analysis of the mineral composition by inductively coupled plasma atomic emission spectrometry (ICP-AES) carried out for the first time allowed the quantification of the mineral elements iron, potassium, phosphorus, magnesium, sodium, copper, calcium, strontium, selenium, and zinc in the aerial part of *Haloxylon scoparium*. The results obtained are presented in Table 1.

Table 1 shows the results of the study of the mineral content of the aerial part of *Haloxylon scoparium*. The analysis of minerals showed that this part of the plant contains high levels of iron, potassium, magnesium, phosphorus, and sodium with values of 60909.00, 27452.10, 10059.90, 1125.39, and 1054.65 mg/kg dry matter, respectively. Copper, calcium, and strontium are present in average amounts, respectively, of the order of 438.93, 313.29, and 280.23 mg/kg of dry matter. Selenium and zinc are present in low levels of 3.00 mg/kg for each.

### 3.2. Phytochemical Study of the Aerial Part of *Haloxylon scoparium*

#### 3.2.1. Yield of Aqueous and Organic Extractions

The aqueous extractions with distilled water carried out hot by decoction and infusion and cold by maceration and the organic extractions hot with Soxhlet with four solvents of different polarities (methanol, ethyl acetate, chloroform, and petroleum ether) and cold by methanol maceration of the aerial part of *Haloxylon scoparium* allowed us to calculate the yield of each aqueous and organic extract. The results obtained are presented in Table 2.

The yields obtained for the aqueous and organic extractions of the aerial part of *Haloxylon scoparium* are presented in Table 2. For the aqueous extracts, the decocted recorded the highest yield followed by the infused and lastly the macerated with percentages of 16, 8, and 5%, respectively. As for the organic extraction, the yields vary according to the solvent used and the extraction method; the methanolic extract prepared with the Soxhlet presents the highest yield of 14.35%, which is higher than the methanolic macerate (10.68%), followed by the chloroform and ethyl acetate extracts which present close values of 2.34 and 2.17%, respectively, the petroleum ether extract comes last with a low yield of 0.89%. In addition, the yield of the decocted aqueous extract (16%) is higher than that of all organic extracts.

#### 3.2.2. Phytochemical Screening

The qualitative evaluation of the chemical composition of the powder of the aerial part of *Haloxylon scoparium* and of the different aqueous and organic extracts prepared from it revealed the presence of the chemical families represented in Table 3.

Phytochemical screening on the powder of the aerial part of the plant showed a strong positive reaction with catechic tannins and alkaloids, a medium positive reaction for flavonoids and saponins, and a weak reaction towards anthracenosides and free quinones.

The aqueous extracts also showed a strong positive reaction for catechic tannins, saponins, and alkaloids except for the aqueous macerate which showed a medium content of saponins. Free quinones are low in the decoctate. For the five organic extracts, catechic tannins were moderately present and alkaloids were strongly present. In addition, the methanolic extract prepared with Soxhlet and the methanolic macerate show a medium reaction with flavonoids, saponins, anthracenosides, and free quinones, and the latter are low in the ethyl acetate and chloroform extracts.

#### 3.2.3. Determination of Polyphenols, Flavonoids, and Catechic Tannins

The results of the phytochemical screening of the aerial part of *Haloxylon scoparium* guided us in the selection of the secondary metabolites to be determined: total phenols, flavonoids, and catechic tannins. The results of the assay are presented in Table 4.

The phytochemical study on the determination of secondary metabolites revealed that the tested extracts contain polyphenols, flavonoids, and catechic tannins (Table 4).

Concerning polyphenols, the aqueous, decocted, infused, and macerated extracts present values of 6.83 ± 0.04, 3.81 ± 0.21, and 3.96 ± 0.07 Ug EAG/mg E, respectively, with a statistically insignificant difference between all aqueous extracts. Polyphenols are more abundant in the methanolic extract prepared in Soxhlet (161.65 ± 1.52 Ug EAG/mg E) and in the methanolic macerate (147.11 ± 6.11 Ug EAG/mg E) with a significant difference, followed, respectively, by ethyl acetate extracts (54.24 ± 2, 70 Ug EAG/mg E) and chloroformic extract (49.42 ± 1.02 Ug EAG/mg E) with a nonsignificant difference. Petroleum ether extract comes in the last position with a polyphenol content of 11.30 ± 1.58 Ug EAG/mg E.

For flavonoids measured in aqueous extracts, the decocted had the highest content (306.59 ± 4.35 Ug EQ/mg E) followed, respectively, by the infused (228.67 ± 10.87 Ug EQ/mg E) and then the macerated (135.78 ± 3.57 Ug EQ/mg E), with a significant difference between them. For the organic extracts, the highest flavonoid content was obtained in the methanolic extract prepared in Soxhlet (612.47 ± 10.10 Ug EQ/mg E) and the methanolic macerate (641.03 ± 7.8 Ug EQ/mg E) with a statistically nonsignificant difference, followed, respectively, by the ethyl acetate extract (416.73 ± 10.18 Ug EQ/mg E) and chloroformic extract (263.25 ± 2.59 Ug EQ/mg E) with a statistically significant difference between the two and lastly the petroleum ether extract (168.3 ± 7.91 Ug EQ/mg E). A significant difference was observed between the decocted and the two organic extracts: the chloroform and petroleum ether extracts expressed by a higher flavonoid content in the decocted compared to the chloroform and petroleum ether extracts.

Concerning the determination of catechic tannins, we found that the aqueous extracts have similar contents; the decoctate has a content of 3.78 ± 0.35 Ug EC/mg E, followed by the infused (1.1 ± 0.13 Ug EC/mg E) and the aqueous macerate (2.25 ± 0.12 Ug EC/mg E), with a nonsignificant difference between the three extracts. As for the organic extracts, the ethyl acetate extract has the highest tannin content (23.69 ± 0.6 Ug EC/mg E) followed by the chloroform extract (21.25 ± 2.25 Ug EC/mg E), petroleum ether extract (7.55 ± 1.18 Ug EC/mg E), and methanolic Soxhlet extract (6.02 ± 0.11 Ug EC/mg E) with a nonsignificant difference, and methanolic macerate comes the last (0.26 ± 0.2 Ug EC/mg E).

### 3.3. *In Vitro* Study of Antidiabetic Activity

The study of the *in vitro* antihyperglycaemic effect of the aqueous and organic extracts of *Haloxylon scoparium* was carried out by the three tests of enzymatic inhibition of *a*-amylase, *a*-glucosidase, and *ß*-galactosidase. The results were expressed as IC50 and are shown in Table 5.

For the *a*-amylase enzyme inhibition test, the results obtained in Table 5 show that the aqueous and organic extracts evaluated present an inhibitory activity with an IC50 which varies between 39096.66 ± 4174.94 ug/mL and 80277.33 ± 7609.97 ug/mL. Concerning the aqueous extracts, the decoctate presents the best inhibitory activity (IC50 = 66855.66 ± 10519.25 ug/mL), followed, respectively, by the infused (IC50 = 78892.33 ± 14448.37 ug/mL) and the macerated (IC50 = 80277.33 ± 7609.97 ug/mL) with a statistically nonsignificant difference between the three extracts. For the organic extracts, ethyl acetate shows inhibitory activity with IC50 = 39096.66 ± 4174.94 ug/mL, followed, respectively, by methanolic macerate (IC50 = 46351 ± 4882.68 ug/mL), chloroformic extract (IC50 = 51261 ± 4786, 07 ug/mL), methanolic extract (IC50 = 56156.33 ± 2580.20 ug/mL), and lastly petroleum ether extract (IC50 = 66601 ± 12217.29 ug/mL) with a statistically insignificant difference between all organic extracts. The aqueous and organic extracts have a lower inhibitory activity for *a*-amylase than the acarbose standard (IC50 = 616.33 ± 5.00 ug/mL).

The study of the inhibition of the enzyme *a*-glucosidase *in vitro* shows that all extracts had high inhibitory activity. For aqueous extracts, decoctate shows an inhibitory activity with IC50 = 181.7 ± 21.15 ug/mL, followed by aqueous macerate (IC50 = 202.1 ± 75.44 ug/mL) and infused (IC50 = 225.44 ± 58.43 ug/mL), respectively; aqueous extracts recorded statistically insignificant difference between them. In addition, the decoctate has a better inhibitory activity compared to acarbose (IC50 = 195 ± 6.12 ug/mL) with a statistically nonsignificant difference. For the organic extracts, the methanolic extract shows an inhibitory activity with IC50 = 193.4 ± 8.57 ug/mL, followed, respectively, by the methanolic macerate (IC50 = 200.86 ± 1.99 ug/mL), ethyl acetate extract (IC50 = 235.9 ± 35.56 ug/mL), chloroform extract (IC50 = 341, 73 ± 13.92 ug/mL), and lastly the petroleum ether extract with an IC50 value of 357.16 ± 2.50 ug/mL; a statistically nonsignificant difference was found between the organic extracts studied and between the latter and acarbose (IC50 = 195 ± 6.12 ug/mL).

The results of the *ß*-galactosidase inhibition test carried out reveal that all the aqueous and organic extracts had inhibitory activity with IC50s ranging between 915.23 ± 68.86 ug/mL and 1984.66 ± 61.65 ug/mL. For the aqueous extracts, infused comes first with an IC50 of 915.23 ± 68.86 ug/mL, followed, respectively, by aqueous macerated (IC50 = 1072.73 ± 369.28 ug/mL) and decocted (IC50 = 1361.66 ± 188.40 ug/mL), with a statistically significant difference between the three extracts. Concerning the organic extracts, the ethyl acetate extract shows the highest inhibitory activity with an IC50 of 1735.66 ± 269.50 ug/mL, followed, respectively, by the chloroform extract (IC50 = 1601.66 ± 107.21 ug/mL), methanolic extract (IC50 = 1735.66 ± 269.50 ug/mL), petroleum ether (IC50 = 1819.66 ± 172.29 ug/mL), and lastly the methanolic macerate (IC50 = 1984.66 ± 61.65 ug/mL). The organic extracts in this test showed a nonsignificant difference between them and a statistically significant difference with quercetin (IC50 = 171.16 ± 5.00 ug/mL).

### 3.4. Antioxidant Activity

The evaluation of the *in vitro* antioxidant activity of the aqueous and organic extracts of the aerial part of *Haloxylon scoparium* was carried out by five tests: H_2_O_2_ scavenging activity test, DPPH radical scavenging test, ABTS radical scavenging test, FRAP test, and PR test. The results obtained are presented in Table 6.

All the extracts studied showed strong antioxidant and free radical scavenging properties, which varied according to the nature of the extract tested and the test used. Moreover, aqueous and organic extracts take the same ranking for all tests; decoctate comes first followed, respectively, by infused and aqueous macerated for aqueous extracts. For the organic extracts, we found the following order for the five tests: methanolic extract > methanolic macerate > ethyl acetate extract > chloroformic extract > petroleum ether extract.

The results of the hydrogen peroxide (H_2_O_2_) scavenging activity reveal that the aqueous extract decoctate has the highest hydrogen peroxide (H_2_O_2_) scavenging capacity (16.21 ± 0.39%), followed by the infused (8.78 ± 0.41%) and the aqueous macerate (4.15 ± 0.43%), respectively, with a significant difference between the three aqueous extracts. For the organic extracts, the methanolic extract shows the highest percentage of hydrogen peroxide (H_2_O_2_) scavenging (20.91 ± 0.27%) with a significant difference with the chloroform, ethyl acetate, and petroleum ether extracts, followed, respectively, by methanolic macerate (7.36 ± 0.09%), ethyl acetate (7.26 ± 0.11%), chloroformic (5.84 ± 0.39%), and lastly petroleum ether extract (5.76 ± 0.4%), with a statistically nonsignificant difference between the four organic extracts. In addition, the hydrogen peroxide scavenging capacity of the decoctate surpassed the methanolic macerated, ethyl acetate, chloroformic, and petroleum ether extracts, as presented in Table 6.

The study of the anti-free radical activity by the DPPH test reveals that all the tested extracts present a considerable anti-free radical activity. Concerning the aqueous extracts, the decoctate showed the highest DPPH scavenging activity with an IC50 of 439.3 ± 7.74 *μ*g/mL, followed, respectively, by the infused (IC50 = 518.96 ± 5.66 *μ*g/mL) and the aqueous macerate (IC50 = 582.8 ± 14.72 *μ*g/mL), with a nonsignificant difference between the three aqueous extracts. For the organic extracts, we found that the methanolic extract shows a very high DPPH radical scavenging power with an IC50 of 39.63 ± 2.03 *μ*g/mL, followed, respectively, by the methanolic macerate (IC50 = 57.87 ± 1.50 *μ*g/mL) with a nonsignificant difference, then by the ethyl acetate extract (IC50 = 62.27 ± 1.82 *μ*g/mL) and chloroform extract (IC50 = 72.00 ± 1.88 *μ*g/mL), with a nonsignificant difference between the two, and lastly petroleum ether (IC50 = 297.8 ± 1.15 *μ*g/mL) which shows a significant difference with all other organic extracts. The free radical scavenging activity of the organic extracts is higher than that of the aqueous extracts, with the exception of the petroleum ether extract, which shows a lower free radical scavenging activity than the decoctate. In spite of the antiradical power of these extracts, it remains significantly lower than the reference standards (ascorbic acid = 0.17 ± 0.02 µg/ml, BHA = 1.59 ± 0.13 µg/ml, and Trolox = 1.75 ± 0.09 µg/ml).

Concerning the ABTS test, we found that the decoctate has the highest antiradical capacity (8.20 ± 0.01 Ug E AA/mg E), higher than the infused (5.14 ± 0.37 Ug E AA/mg E) and the aqueous macerate (3.99 ± 0.26 Ug E AA/mg E); however, they present a statistically nonsignificant difference between them. For the organic extracts, we noticed that the methanolic extract has the highest antiradical capacity (50.75 ± 0.72 Ug E AA/mg E), followed by the methanolic macerate (47.71 ± 1.21 Ug E AA/mg E) with a nonsignificant difference, then by the ethyl acetate extract (39.74 ± 1.41 Ug E AA/mg E) and chloroformic extract (36.99 ± 1.34 Ug E AA/mg E) with a nonsignificant difference, and lastly petroleum ether extract (1.72 ± 0.53 Ug E AA/mg E) with a statistically significant difference with all the organic extracts (Soxhlet methanolic, methanolic macerated, chloroformic, and ethyl acetate). The organic extracts in this test have a higher free radical scavenging activity than the aqueous extracts with a significant difference, except for the petroleum ether extract, which has a lower free radical scavenging capacity than the aqueous extracts with a significant difference with the decoctate and a nonsignificant difference with the infused and aqueous macerate.

The results of the antioxidant activity by the FRAP test reveal that the decoctate comes first with a reducing capacity of 37.66 ± 1.29 Ug E T/mg E, followed, respectively, by the infused (27.94 ± 1.08 Ug *E* T/mgE) with a nonsignificant difference and the aqueous macerate (17.81 ± 3.50 Ug E T/mg E) with a significant difference with the decoctate and a nonsignificant difference with the infused.

Concerning the organic extracts, the methanolic extract presents the highest reducing capacity of ferric iron (Fe3+) to ferrous iron (Fe2+) with a value of 163.37 ± 1.52 Ug E T/mg E, followed, respectively, by the methanolic macerate, ethyl acetate, chloroformic, and petroleum ether extracts with values of 124.08 ± 6.97, 106.14 ± 5.2, 85.02 ± 2.96, and 24.51 ± 0.53 Ug *E* T/mg E, respectively. Statistical analysis showed a significant difference between all organic extracts.

According to the results obtained, the aqueous extracts also show a higher reducing power in this test than the petroleum ether extract with a statistically nonsignificant difference between the 3 aqueous extracts: decocted (37.66 ± 1.29 Ug E T/mg E), infused (27.94 ± 1.08 Ug E T/mg E), and macerated (17.81 ± 3.50 Ug E T/mg E).

The results of the reducing power test show that the decoctate has a higher reducing capacity than the infused and aqueous macerated extracts, which are, respectively, in the order of 21.89 ± 1.04, 14.09 ± 0.74, and 6.63 ± 0.40 Ug E AA/mg E with a nonsignificant difference.

For organic extracts, methanolic extract and methanolic macerate show the highest reducing power of 116.18 ± 8.19 and 110.11 ± 7.47 Ug E AA/mg E, respectively, with a nonsignificant difference between the two extracts, followed by ethyl acetate extract (79, 27 ± 4.78 Ug E AA/mg E) and chloroformic extract (59.35 ± 0.65 Ug *E* AA/mg E) with a nonsignificant difference between them and finally petroleum ether extract (0.96 ± 0.3 Ug E AA/mg E) which shows a significant difference with all organic extracts. The aqueous extracts have a higher iron reduction capacity than the petroleum ether extract with a statistically nonsignificant difference.

### 3.5. Principal Component Analysis (PCA)

The principal component analysis (PCA) allowed us to highlight the correlation between the aqueous and organic extracts and their antioxidant capacity evaluated by the different tests and the correlation between these extracts and their chemical compound content.

The objective of the PCA carried out on eight individuals divided into three aqueous extracts and five organic extracts of the aerial part of *Haloxylon scoparium* was to highlight the possible correlations existing between the individuals and the variables tested, in relation to eight variables represented the content of chemical compounds (total polyphenols, flavonoids, and catechic tannins) and, on the other hand, in relation to the *in vitro* inhibitory activity of *a*-amylase, *a*-glucosidase, and *ß*-galactosidase and with the five tests used for the evaluation of antioxidant activity: H_2_O_2_, DPPH, ABTS, FRAP, and PR.

#### 3.5.1. Correlation Matrix

Principal component analysis (PCA) showed that the DPPH test is highly positively correlated with the ABTS (*r*^2^ = 0.9716), PR (*r*^2^ = 0.9333), and FRAP (*r*^2^ = 0.9495) tests. The ABTS test is highly positively correlated with the FRAP (*r*^2^ = 0.9713) and PR (*r*^2^ = 0.9809) tests. The FRAP and PR tests have a high positive correlation with each other of *r*^2^ = 0.9845.

Polyphenol content is highly positively correlated with all antioxidant activity tests except the H_2_O_2_ test (DPPH, *r*^2^ = 0.8549; ABTS, *r*^2^ = 0.8944; FRAP, *r*^2^ = 0.9372; and PR, *r*^2^ = 0.9429). Flavonoid content was also strongly positively correlated with the tests (DPPH, *r*^2^ = 0.7909; ABTS, *r*^2^ = 0.8567; FRAP, *r*^2^ = 0.8730; and PR, *r*^2^ = 0.8983). In addition, total polyphenols showed a high positive correlation with flavonoid content (*r*^2^ = 0.9416) (Table 7).

The inhibitory activity of *a*-amylase was highly positively correlated with antioxidant activity assays: DPPH (*r*^2^ = 0.8094), ABTS (*r*^2^ = 0.8237), FRAP (*r*^2^ = 0.8115), and PR (*r*^2^ = 0.8508); *a*-amylase was highly positively correlated with total polyphenol (*r*^2^ = 0.7721) and flavonoid (*r*^2^ = 0.7162) content. The *in vitro* inhibitory activity by *a*-glucosidase and *ß*-galactosidase is moderately positively correlated with the H_2_O_2_ antioxidant activity test with values of *r*^2^ = 0.4885 and *r*^2^ = 0.0412, respectively.

#### 3.5.2. Graphical Representation of the Principal Component Analysis (PCA)

According to the principal component analysis (PCA) (Figure 2), the two main axes (F1 and F2) describe 83.39% of the total variance of the observations. Therefore, the interpretations made from this analysis will be highly significant. This analysis allowed us to discriminate three groups:

  Group 1: it contains the methanolic extract and the methanolic macerate, presents the highest contents of total polyphenols and flavonoids, and also expresses a better antiradical activity via the DPPH, ABTS, and H_2_O_2_ tests and a high reducing power via the FRAP and PR tests. In addition, both extracts show inhibitory activity of *a*-amylase and *a*-glucosidase enzymes.
  Group 2: it includes the chloroformic extract which has high tannin content and intermediate *in vitro* antioxidant and antidiabetic activity.
  Group 3: it consists of the organic ethyl acetate extract which expresses a high content of catechic tannins and presents a strong inhibitory activity of the enzymes *ß*-galactosidase and *a*-amylase. This group also includes the petroleum ether extract and the aqueous extracts, decocted, infused, and macerated, which have low levels of phenolic compounds, but are rich in flavonoids and have moderate antioxidant and antidiabetic activity *in vitro.*

## 4. Discussion

### 4.1. Study of the Mineral Composition of the Aerial Part of *Haloxylon scoparium*

The results of the mineralogical analysis reveal the richness of the aerial part of *Haloxylon scoparium* in minerals, with a high content of iron, potassium, and magnesium and a significant content of phosphorus, sodium, and copper. Calcium and strontium are present at medium levels. The aerial part of *Haloxylon scoparium* is characterised by its richness in minerals that could be responsible for its biological activities. From the mineralogical study, we have highlighted the presence of a high content of Fe, K, P, Na, Cu, Mg, Ca, and Sr compared to those obtained in a recent work carried out by Boulfia and his collaborators (Fe (33552), K (1843.14), P (756.36), Na (439.65), Cu (303.9), Mg (272.37), and Ca (20.55) mg/kg of plant material), and the antioxidant capacity that we recorded is higher than that obtained by Boulfia his collaborators for the ethanolic extract with Soxhlet [28], which could confirm that some minerals may be responsible for the antioxidant capacity of the aerial part of *Haloxylon scoparium*. In this sense, a study conducted on *Phoenix dactylifera* fruits showed a high correlation between antioxidant activity and mineral composition; K content is highly correlated with the FRAP test (*r*^2^ = 0.800) and with the H_2_O_2_ test (*r*^2^ = 0.889) [29]. This is in agreement with our results on antioxidant activity for both tests. Minerals play a crucial role in antioxidant activity; according to Grela et al., the antioxidant activity is attributed to mineral components such as copper, manganese, and iron [30]. Furthermore, an imbalance of mineral elements would change the content of flavonoids considered as a proven antioxidant compound [31]. Some antioxidant enzymes require metal ions for their activity; other metals have been directly classified as antioxidants [32]. Many antioxidant defence pathways are dependent on micronutrients. Some minerals are components of antioxidant enzymes: superoxide dismutase depends on Mn, Cu, and Zn; catalase depends on Fe, and glutathione peroxidase on Se [33]. Minerals may also be responsible for antidiabetic activity; several minerals are involved in glucose metabolism such as Ca, K, Mg, and Na [34]; in addition, several studies have shown the relationship between oxidative stress and the development of diabetes. An increase in oxidative stress can cause an alteration of the insulin signalling pathway, either by a decrease in glucose capture by insulin-sensitive tissues or by an increase in hepatic glucose production, which leads to the development of insulin resistance and subsequently noninsulin-dependent diabetes [35].

### 4.2. Phytochemical Study

#### 4.2.1. Yield of Aqueous and Organic Extracts

The results of the phytochemical study show that among the aqueous extracts, the decoctate presented a better yield in comparison with the infused and macerated with percentages of 16%, 8%, and 5%, respectively. These extracts were prepared with distilled water but at different temperatures, which means that the amount of extractable material from the aerial part of *Haloxylon scoparium* increases with the increase of temperature during the aqueous extraction.

For the organic extracts, the yields vary according to the polarity of the solvent used and the method and modality of extractions; the yield of the methanolic extract prepared with Soxhlet is higher than that of the methanolic macerate with 14.35 and 10.68%, respectively. This variation is probably due to the temperature used, the extraction time, and the technique used. The Soxhlet methanolic extract has the highest amount of extracted material, which suggests that the use of methanol as an organic solvent may be suitable for the extraction of natural chemical compounds from the studied part of the plant.

The extraction yield varies depending on the plant species, the part used in the extraction, the harvesting period, the type of soil, the climate, the geographical position, the drying conditions including the duration, the form of the plant material (powder or fragments), the nature of the solvent used in the extraction and its polarity and the extraction conditions: temperature, extraction duration, solvent/plant material ratio.

According to Jurinjak Tušek et al., the extraction yield of the Asteraceae family increases by increasing the extraction temperature [36]. According to Kwon and Chung, the maximum extraction yield of *Curcuma longa* was obtained at 135°C/5 min with a ratio of water: ethanol (50 : 50, v/v) as extraction solvent [37]. Wu et al. also found that temperature, extraction time, and solvent/plant material ratio affect the yield of *Ziziphus jujuba* [38].

In 2012, Lamchouri and his collaborators conducted a phytochemical study on the aerial part of *Haloxylon scoparium* and obtained yields of 10.50% for the decoctate, 10.47% for the Soxhlet methanolic extract, and 10.00% for the methanolic macerate. These yields are lower than those obtained in our study [7]. This variation could be explained by the difference in the harvesting period which was between March and April in 2012 and by the plant material/solvent ratio which was 20 g of plant material/250 ml of each solvent for the 2012 study. In contrast, the 2019 harvest was done in July, and the plant material to solvent ratio was 20 g plant material/200 ml of each solvent.

According to work conducted on other plants from the region of Taza, Morocco, in our laboratory under the same operating conditions, Bouabid and collaborators found that the best yields are obtained with polar solvents and that hot extraction gives the higher yields when compared to cold extraction for aqueous and organic extracts of the underground part of *Atractylis gummifera* [12]. Senhaji and her collaborators found that the aqueous macerate and hot methanolic extract of *Ajuga iva* had the high yield of 13.31% and 9%, respectively. Similarly, aqueous macerate and methanolic extract prepared hot in Soxhlet from the aerial part of *Anabasis aretioides* of the family Chenopodiaceae show the highest yield of 3.41% and 3.39%, respectively [15,16]. Boulfia and his collaborators found that the hot-prepared ethanolic extract and the decoctate of *Juglans regia* had the highest yields of 22.04% and 14% [14].

#### 4.2.2. Phytochemical Screening

The phytochemical screening carried out on the powder of the aerial part of *Haloxylon scoparium* and on the aqueous and organic extracts prepared from it allowed us to highlight the presence of different secondary metabolites; the plant is highly rich in catechic tannins and alkaloids that are contained in the powder of the plant material and in all the aqueous and organic extracts. Our results are in agreement with other works that indicated the richness of *Haloxylon scoparium* in alkaloids; Zerriouh and collaborators reported that the aerial part of *Hammada scoparia* collected in Algeria contains the alkaloids [39]. In addition, Jarraya and collaborators described the isolation and structural elucidation of N-methylisososaloline extracted from *Haloxylon scoparium* leaves collected in Tunisia [40].

The plant material and the aqueous and organic extracts contain catechic tannins, which are known to possess multiple pharmacological properties, antiinflammatory [41], antidiabetic [42], antimicrobial, and antiviral activity [43]. In this sense, a study conducted in our laboratory by Lamchouri and collaborators showed that the *Staphylococcus aureus* strain presented a good sensitivity of 7–12 mm to ethyl acetate extract of *H. scoparium* [7].

Saponins are strongly present in aqueous extracts, mainly decocted and infused, and moderately present in methanolic extract and its macerate; saponins are best extracted at high temperature. According to Nafiunisa and collaborators, the amount of extracted saponin increases with increasing extraction temperature [44]. Concerning flavonoids, the reaction of their detection was moderately positive at the level of the three aqueous extracts, the methanolic extract prepared with Soxhlet, and the methanolic macerate. Quinones and anthracenosides were present in the decoctate and the methanolic, methanolic macerated, ethyl acetate, and chloroform extracts.

A study done by Zerriouh and collaborators in Algeria showed that the aqueous extract of the aerial part of *Hammada scoparia* is devoid of flavonoids but contains the alkaloids and saponins, while the methanolic extract prepared in Soxhlet contains flavonoids, alkaloids, and tannins [39]. Furthermore, a study done by Bourogaa and collaborators in Algeria revealed the presence of flavonoids and alkaloids, while sterols and quinones are absent from the aqueous extract of *H. scoparia* leaves [45].

In the same operating conditions, works carried out on plants collected in the same region as *Haloxylon scoparium* in our laboratory by Senhaji and collaborators, Bouabid and collaborators, and Boulfia and collaborators revealed that phytochemical screening showed the presence of catechic tannins, saponins, and sterols in the aerial part of *Anabasis aretioïdes* which belongs to the same Chenopodiaceae family as our *H. scoparium* plant [16]. The underground part of *Atractylis gummifera* is characterised by the presence of tannins and flavonoids [12], and the bark of *Juglans regia* is rich in catechic tannins, flavonoids, anthraquinones, and free quinones [14]. Catechic tannins, flavonoids, saponins, and sterols are present in the aerial part of *Ajuga iva* [15].

#### 4.2.3. Determination of Total Polyphenols, Flavonoids, and Catechic Tannins

The quantitative analysis of phenolic compounds in the aerial part of *Haloxylon scoparium* showed that all extracts are richer in total polyphenols, flavonoids, and tannins.

The aqueous extracts show low amounts of total polyphenols, and the decoctate comes first with a value of 6.83 ± 0.04 Ug EAG/mg E, followed by the aqueous macerate (3.96 ± 0.07 Ug EAG/mg E) and the infused (3.81 ± 0.21 Ug EAG/mg E) with a statistically nonsignificant difference. For the organic extracts, the total polyphenols are better extracted by methanol; moreover, the polyphenol content in the Soxhlet methanolic extract exceeds that of the methanolic macerate with a significant difference. This variation may be due to the factor of the technique used; in fact, the Soxhlet extraction allows the total exhaustion of the plant material through the successive repetition of the extraction cycles at a temperature of 64.7°C for 7 hours, which allows the maximum extraction of total polyphenols. The organic extracts have the highest content of total polyphenols compared to the aqueous extracts. The richness of organic extracts compared to aqueous extracts could be explained by the capacity of organic solvents to extract bioactive molecules. According to Toledo-Guillén and collaborators, extraction by organic solvents is more efficient to obtain bioactive compounds [46].

In the same operating conditions, the work carried out in our laboratory by Senhaji and her collaborators on a plant of the same family showed that the decoctate and the aqueous macerate have high contents of total polyphenols (1.78 ± 0.003 and 0.92 ± 0.03 mg EAG/g E); moreover, ethyl acetate is the recommended solvent for the extraction of polyphenols from the aerial part of *Anabasis aretioïdes* [16]. Another study conducted by Bouabid and her collaborators revealed that polyphenols are very abundant in the methanolic macerate of *Atractylis gummifera* (102.88 ± 1.38 mg EAG/g E) [13]. According to Senhaji and her collaborators, decoction is the mode that allows a high extraction of polyphenols (3.75 ± 0.02 EAG/g E) from the aerial part of *Ajuga iva* subsp. pseudoiva [15]. Boulfia and his collaborators found that the acetone macerate of *Juglans regia* bark is the richest in phenolic compounds (327.972 ± 0.06 *µ*g EAG/mg E) [14].

As for the flavonoids, they are clearly abundant in all the aqueous extracts of the aerial part of *Haloxylon scoparium*; the decoctate comes first with a content of 306.59 ± 4.35 Ug EAG/mg E, followed, respectively, by the infused (228.67 ± 10.87 Ug EAG/mg E) and the macerated (135.78 ± 3.57 Ug EAG/mg E), with a significant difference between the three aqueous extracts.

The flavonoid content of the organic extracts increased with the degree of polarity of the organic solvents used for extraction; this could be explained by the variation in the solubility of phenolic compounds depending on the polarity of the extraction solvent used. Furthermore, in the present study, the highest content was obtained in the methanolic extract prepared hot in Soxhlet and methanolic macerate with a statistically insignificant difference; methanol could be recommended for the extraction of flavonoids.

However, the content recorded by the decoctate exceeds that of the chloroform and petroleum ether extracts, which could be explained, on the one hand, by the high polarity of water compared to chloroform and petroleum ether and, on the other hand, by the high polarity and water solubility of the flavonoids present in the aerial part of *Haloxylon scoparium*. In addition, the high temperature could favour the solubility of the flavonoids contained in the plant. Tan and Kassim conducted a phytochemical study on the plant *R. apiculata* and found that the flavonoid content increases with increasing temperature and that the amount of flavonoids extracted by water at 90°C exceeds that of ethanolic and acetone extracts [47].

According to a study conducted in Algeria, Ziani and collaborators found that the infused aerial part of *Haloxylon scoparium* has a polyphenol content of 230 ± 8 mg GAE/g E and a flavonoid content of 56 ± 1 mg CE/g E [48]. Another study conducted in Algeria by Chaouche and collaborators revealed that the hydromethanolic extract of the aerial part of *H. articulatum* has low contents of total polyphenols and flavonoids compared to the content of our methanolic extract [49]. Another Tunisian study was conducted by Bouaziz and collaborators [50] and revealed that the total polyphenol content of the methanolic extract of *H. scoparium* leaves is 59.75 ± 1.80 mg GAE/g, which is low compared to that of our methanolic extract. The difference in these results can be explained by factors related to the harvesting of the plant such as geographical location, harvesting season, maturity stage of the harvested plant, part of the plant harvested, and factors related to the experiment such as plant/solvent ratio, temperature, and extraction time. These same deductions and conclusions were found from several works carried out on several plants from the same region of Taza, Morocco, in our laboratory [13–16]. Indeed, Bouabid and collaborators found that the methanolic macerate of the aerial part of *Atractylis gummifera* has a flavonoid content of the order of 17.25 ± 0.06 mg ER/g E [13]. Boulfia and collaborators found that the acetone macerate of *Juglans regia* bark contains the highest flavonoid content (1267.981 ± 2.911 *µ*g EQ/mg E) [14]. According to Senhaji and collaborators, the ethyl acetate extract of *Ajuga iva* is the mode that allows high flavonoid extraction (22.40 ± 0.36 mg ER/g E) [15]. In contrast, a phytochemical study conducted by Senhaji and collaborators on the aerial part of *Anabasis aretioides*, which belongs to the Chenopodiaceae family, showed a complete absence of flavonoids [16].

Concerning the tannin content, it varies according to the extracts analysed. For the aqueous extracts, tannins are poorly present, which could be explained by the low solubility of condensed tannins in water. According to Gun'ko et al., tannins are less soluble in water due to the low surface area accessible to water molecules [51]. In addition, the large value recorded for aqueous extracts was for the decoctate (3.78 ± 0.35 Ug EC/mg E), which could be due to the ability of hot water to extract condensed tannins. These results agree with those obtained by Tan and Kassim on *R. apiculata*, who found that condensed tannins are more soluble in water at high temperatures [47]. A study done in Algeria by Chaouche and collaborators revealed that the hydromethanolic extract of the aerial part of *H. articulatum* presents a content of 9.98 ± 1.6 mg EC/g dry matter [49].

For the organic extracts, the highest tannin value was recorded by ethyl acetate (23.69 ± 0.6 mg EC/g E) and chloroform (21.25 ± 2.25 mg EC/g E) with a statistically nonsignificant difference, followed by petroleum ether and Soxhlet methanolic extracts, respectively. However, the methanolic macerate showed low tannin content. The difference obtained between the two extracts (methanolic extract and methanolic macerate) prepared with the same methanolic solvent allows us to confirm that hot extraction allows better extraction of tannins.

These differences could be due to the properties of the tannins in the test portion to solubilise in the solvents used. According to Bele et al., tannins are generally divided into hydrolysable and condensed tannins; the former can be hydrolysed by weak acids and bases to produce carbohydrates and phenolic acids. However, condensed tannins are not susceptible to hydrolytic cleavage [52].

As a comparison, work carried out under the same operating conditions in our laboratory by Bouabid and collaborators revealed that the methanolic macerate of *Atractylis gummifera* is richer in catechic tannins (144.09 ± 3.96 mg EC/g E) [13]; acetone macerate of *Juglans regia* bark is rich in tannins (38.056 ± 1.886 *µ*g EC/g E) [14]; aqueous macerated of *Ajuga iva* allows a high extraction of catechic tannins (15.49 ± 0.17 mg EC/g E) [15]; and ethyl acetate extract of the aerial part of *Anabasis aretioides* of the Chenopodiaceae family has the highest tannin content (46.46 ± 0.67 mg EC/g E) [16].

### 4.3. *In Vitro* Study of Antidiabetic Activity

The *in vitro* antihyperglycaemic effect of aqueous and organic extracts of *Haloxylon scoparium* carried out by the enzymatic inhibition tests of *a*-amylase, *a*-glucosidase, and *ß*-galactosidase showed that all the extracts possess inhibitory activity with different degrees. The decoctate had an inhibitory effect against *a*-amylase with IC50 = 66855.66 ± 10519.25 ug/mL, which is higher than those of the infused and aqueous macerate, which could be explained by the ability of the high temperature to extract molecules that have the capacity to inhibit *a*-amylase. Ethyl acetate shows the best *a*-amylase inhibitory activity compared to other organic extracts; this *a*-amylase inhibitory activity is probably related to the presence of phenolic compounds in this plant. Hanhineva and collaborators reported that flavonoids, phenolic acids, and tannins inhibit the activity of enzymes such as *a*-amylase and *a*-glucosidase [53]. This is proved by the phytochemical study we performed, which revealed that ethyl acetate extract has the high content of catechic tannins (23.69 ± 0.6 Ug EC/mg E) among other organic extracts.

For the *a*-glucosidase assay, all products showed a very high activity compared to the reference standard. For the aqueous extracts, the decoctate showed an inhibitory activity with IC50 = 181.7 ± 21.15 ug/mL, which is higher than those obtained by the infused (IC50 = 225.44 ± 58.43 ug/mL) and the aqueous macerate (IC50 = 202.1 ± 75.44 ug/mL). The decoctate shows a significantly higher activity than acarbose (IC50 = 195 ± 6.12 ug/mL) with a statistically nonsignificant difference. This effect may be due to the presence of secondary metabolites extracted at high temperature. For organic extracts, the inhibitory activity of *a*-glucosidase was recorded according to this order: methanolic extract > methanolic macerate > ethyl acetate extract > chloroformic extract > petroleum ether extract, which shows that the inhibitory activity varies according to the polarity of the solvents used for extraction; a recent study carried out in Japan by Dirar and collaborators showed that polar extracts of *G. senegalensis* exhibited better inhibitory activity on *a*-glucosidase [54].

The results of enzymatic inhibition of *ß*-galactosidase of the aqueous extracts show that the infused comes first, followed, respectively, by the aqueous macerated and lastly the decocted which could be explained by the nature of the molecules responsible for the activity which are degradable at high temperature at a longer duration. For the organic extracts, ethyl acetate extract presents the best inhibitory activity with an IC50 of 1601.66 ± 107.21 ug/mL followed, respectively, by chloroformic extract (IC50 = 1707.66 ± 12.99 ug/mL), methanolic extract (IC50 = 1735.66 ± 269.50 ug/mL), petroleum ether extract (IC50 = 1819.66 ± 172.29 ug/mL), and finally methanolic macerate (IC50 = 1984.66 ± 61.65 ug/mL). These results are in agreement with those obtained by El Omari and collaborators on *A. longa* who found that the ethyl acetate fraction had the highest inhibitory activity against *ß*-galactosidase (12.70 ± 1.27%) and the methanolic fraction showed moderate inhibition of *ß*-galactosidase (2.05 ± 1.22%) [55]. The degree of inhibitory activity of aqueous and organic extracts of *Haloxylon scoparium* varies from test to test; according to Chiba and collaborators the differences between the enzymes *a*-amylase and *ß*-galactosidase is due to structural differences related to the origin of the enzymes [56].

The antidiabetic activity could be not only due to the phenolic compounds, flavonoids, and catechic tannins but also due to the mineral compounds contained in the studied part: calcium, potassium, magnesium, and sodium are involved in the glucose metabolism [34]. Calcium improves glucose tolerance. In case of deficiency, its metabolism may be directly involved in the occurrence of noninsulin-dependent diabetes [57]. Potassium is involved in the production of glycogen and the secretion of hormones, particularly insulin. Its deficiency is responsible for glucose intolerance [58]. Magnesium is an enzyme activator; it increases insulin secretion and facilitates the use of glucose [59]. The aerial part of *Haloxylon scoparium* is rich in mineral elements (Fe, K, Mg, P, Na, Cu, Ca, and Sr) that can contribute to glucose metabolism. A recent study conducted by Boulfia and his collaborators found that *Juglans regia* L. bark has several minerals (Fe (19849.8), K (3487.8), Mg (2631.03), and P (691.02) mg/kg); these values remain lower than those found by our study. Similarly the antidiabetic activity that we obtained is higher compared to the ethanolic extract of *Juglans regia* L. bark for the *a*-amylase (IC50 = 7806.33 ± 85.08 *μ*g/mL) and *a*-glucosidase (IC50 = 488.83 ± 36.34 *μ*g/mL) inhibition tests [60]. Therefore, a richness of the aerial part of *Haloxylon scoparium* in mineral compounds could explain the hypoglycemic effect of its extracts.

An *in vitro* antihyperglycaemic study conducted by Bouabid and her collaborators in our laboratory under the same experimental conditions on extracts prepared at different polarity from *Atractylis gummifera* harvested in the region of Taza, Morocco, showed that the methanolic macerate presents the highest inhibitory activity for the three enzymes *a*-amylase (IC50 = 557 ± 0.013 ug/mL), *a*-glucosidase (IC50 = 743 ± 0.017 ug/mL), and *ß*-galactosidase(IC50 = 2443 ± 0.071 ug/mL) [12].

### 4.4. *In Vitro* Antioxidant Activity

The study showed that the aqueous and organic extracts studied have an interesting antioxidant power, mainly those prepared by the solvents methanol, ethyl acetate, and chloroform for the organic extracts and the decoctate for the aqueous extracts.

#### 4.4.1. Hydrogen Peroxide Scavenging Activity

The results of the activity of the aqueous extracts obtained reveal that the decoctate has the best hydrogen peroxide scavenging activity compared to the infused and the aqueous macerate which can be attributed to its high flavonoid content. According to Ghedira, the best described property of flavonoids is their antioxidant activity and their ability to neutralise free radicals through their highly reactive hydroxyl group (C3-OH) [61].

For the organic extracts, the hydrogen peroxide (H_2_O_2_) blocking activity revealed that the methanolic extract has the highest free radical scavenging capacity with a value of 20.91 ± 0.27%, which is in agreement with the high polyphenol and flavonoid contents of this extract. However, the methanolic macerated extract shows a lower free radical scavenging activity against hydrogen peroxide, but very close to those of ethyl acetate, chloroformic, and petroleum ether extracts with a statistically nonsignificant difference.

With the hydrogen peroxide (H_2_O_2_) blocking test, we noted a strong capacity to neutralise hydrogen peroxide of the methanolic extract and the aqueous decoctate superior to that of the reference standard ascorbic acid. Thus, we can deduce that the molecules responsible for hydrogen peroxide scavenging are best extracted by high polarity and high temperature solvents. Furthermore, the hydrogen peroxide scavenging capacity may be due to the richness of the studied part in mineral compounds (Fe, K, Mg, P, Na, Cu, Ca, and Sr); this is in agreement with a study conducted on *Phoenix dactylifera* fruits which showed a high correlation between the H_2_O_2_ test and K content (*r*^2^ = 0.889) [29].

In the same operating conditions, the phytochemical study conducted on *Atractylis gummifera* revealed that the best antioxidant activity via the H_2_O_2_ test (19.24 ± 1.102%) was obtained by the methanolic macerate [13]. Furthermore, the acetone-macerated extract of *Juglans regia* showed a high antioxidant activity by the H_2_O_2_ test (24.13 ± 1.81%) [14]. In addition, a phytochemical study conducted on *Ajuga iva* showed that the methanolic macerate had an antioxidant activity of 22.17 ± 0.30% for the H_2_O_2_ test [15]. Another phytochemical study conducted on *Anabasis aretioides* which belongs to the same family of *Haloxylon scoparium* showed that the aqueous macerate exhibits the highest antioxidant activity for the H_2_O_2_ test (7.84 ± 0.44%) [16].

#### 4.4.2. DPPH Radical Scavenging Activity

According to the results obtained with the DPPH test, the aqueous extracts present relatively high IC50 values which indicates a low antiradical power in contrast to the organic extracts which present a high antiradical power; we noticed that the IC50 values of the organic extracts range from 39.63 ± 2.03 for the methanolic extract to 297.8 ± 1.15 *μ*g/mL for the petroleum ether extract. A strong free radical scavenging capacity is noted for the methanolic extract prepared under hot Soxhlet conditions, the aqueous macerate, and the ethyl acetate extract with a statistically nonsignificant difference. This is probably due to the richness of these extracts in phenolic compounds including total polyphenols, tannins, and flavonoids, which gives a better antiradical activity. These results are in agreement with the contents of quantified phenolic compounds. Similarly, Turkmen and collaborators found a significant correlation between total polyphenols extracted from black tea and free radical scavenging activity via the DPPH test [62]. Additionally, the antiradical activity of the different extracts studied could be due to the mineralogical richness of *Haloxylon scoparium*. According to Tamuly and his collaborators, there is a positive correlation between the K content and the capacity to trap the free radical DPPH [63].

For the comparative purposes, the antiradical power of our methanolic and methanolic macerated extract are stronger than that of the hydromethanolic extract of the aerial part of *Haloxylon scoparium* tested by Chaouche and collaborators in Algeria (IC50 = 6.32±0.25 mg/mL) [49]. Furthermore, our extracts are more potent compared to a study done by Miguel and collaborators in Portugal on the hydroalcoholic extract of the aerial part of *H. articulatum* (IC50 = 1.867 ± 0.061 mg/ml) [64]. The results obtained by Bouaziz and collaborators with the aqueous extract of *H. scoparia* leaves from Tunisia showed a high antiradical activity with an IC50 value in the range of 28 ± 0.70 *μ*g/mL [50].

In the same conditions of operation, phytochemical studies recently conducted in our laboratory with the DPPH test showed that the best antioxidant activity of *Atractylis gummifera* was obtained with the aqueous macerate which was found to be the most active (IC50 = 2.78 ± 1.03 *μ*g/mL) [13]. Moreover, the acetone macerate of *Juglans regia* has the highest antioxidant activity (IC50 = 5.573 µg/ml) [14]. In addition, the methanolic extract of *Ajuga iva* is the most active (IC50 = 78.40 ± 5.24 µg/mL) [15]. Another phytochemical study conducted on the aerial part of a plant of the Chenopodiaceae family, *Anabasis aretioides*, indicated that the methanolic macerate has the high level of antioxidant activity (IC50 = 52.91 ± 0.24 *µ*g/ml) [16].

#### 4.4.3. Equivalent Antioxidant Capacity of Trolox (TEAC or ABTS)

According to the ABTS test, we noticed that the aqueous extracts present an antiradical activity with a nonsignificant difference; this could be explained by the composition of these extracts in polyphenols and catechic tannins with statistically nonsignificant values.

The results also show that the organic extracts present a remarkable antioxidant effect towards the ABTS radical. The best antioxidant activity to trap the ABTS free radical was obtained by the methanolic extract (50.75 ± 0.72 Ug E AA/mg E) and the methanolic macerate (47.71 ± 1.21 Ug E AA/mg E) with a statistically nonsignificant difference. This activity is correlated with their high content of total polyphenol and flavonoids compared to the other extracts.

In addition, the decoctate presents a significant antiradical activity among the aqueous extracts, which is also higher than that of the organic petroleum ether extract; this could be explained, on the one hand, by the variability of the solubilisation capacity of the ABTS^•+^ radical in the organic and aqueous media and, on the other hand, by the richness of the decoctate in flavonoids. Bhouri and collaborators reported that flavonoids have a potential activity towards the ABTS^•+^ radical due to the fact that they are rich in hydroxyl groups and therefore stabilise the reactive oxygen species by reaction with the reactive compound of the radical. Because of the high reactivity of the hydroxyl group of flavonoids, the radicals are inactivated [65]. Moreover, the free radical scavenging activity of the ABTS test could be due to the neutralisation of the ABTS^•+^ radical by some minerals contained in the plant; according to Gordon, K plays a role in the activation of enzymes that promote the biosynthesis of flavonoids and phenolic compounds, the latter being endowed with an important antioxidant power [66]. Furthermore, in a study conducted by Chaouche and collaborators in Algeria on the hydromethanolic extract of the aerial part of *Haloxylon articulatum* with the ABTS assay, they obtained an IC50 value in the order of 40.94 ± 3.30 mg/mL [49].

With the same operating conditions, Bouabid and collaborators found that the methanolic macerate of *Atractylis gummifera L* has given the strongest antioxidant activity in the ABTS test (122.6 ± 0.63 mg TE/g E) [13]. Boulfia and collaborators found that the acetone macerate showed the most strong antioxidant activity in the ABTS test (602.29 ± 0.34 *μ*g ET/mg E) [14]. In addition, Senhaji et al. conducted a study on *Ajuga iva* under the same operating conditions as our work and found that the chloroform extract was the most active in the ABTS test (27.33 ± 1.08 *µ*g TE mg-1E) [15]. Another study conducted on a plant of the Chenopodiaceae family, *Anabasis aretioides*, showed that the methanolic macerate exhibited the most high level of antioxidant activity in the ABTS test (48.99 ± 1.316 *µ*g TE/mg E) [16].

#### 4.4.4. Ferric Reducing Antioxidant Power (FRAP) Assay

For the FRAP test, all extracts showed reducing power. The aqueous, decocted and infused extracts show high iron reducing capacity with a statistically insignificant difference, while the aqueous macerate exerts a less remarkable reducing activity with a significant difference to the decocted and a nonsignificant difference to the infused. The compounds responsible for iron reduction are present in the aqueous extracts prepared at high temperature. This activity of the aqueous extract is probably due to the presence of a high level of flavonoids demonstrated in the secondary metabolite assay. Our results are in agreement with a recent work by Hmidani and collaborators on *Thymus atlanticus*; they found that the decoctate has a significant reducing power (19.06 ± 0.54 *μ*mol Trolox E/1 g DM) than the aqueous macerate (4.37 ± 0.24 *μ*mol Trolox E/1 g DM) [67].

Concerning the organic extracts, the reducing power increases with the increase of the polarity of the solvent used; the methanolic extract, the methanolic macerated extract, and the ethyl acetate extract present the highest powers to convert ferric (Fe^3+^) into ferrous (Fe^2+^) with a significant difference. This could be related to the high amount of total polyphenols and flavonoids in these extracts. In addition, the chloroformic extract shows an average but higher reducing capacity than the petroleum ether extract with a significant difference; the latter contains lower contents of total polyphenols (11.30 ± 1.58 Ug EAG/mg E) than the other organic extracts. This result is in agreement with a study done by Saffarzadeh-Matin and Khosrowshahi in which they found a correlation between the FRAP test and the content of phenolic compounds and flavonoids contained in the ethanolic extract of *Punica granatum* harvested in Iran [68]. In addition, according to Mohamed and his collaborators, the FRAP test of date fruits showed a highly significant positive correlation with K (*r*^2^ = 0.800) and Ca (*r*^2^ = 0.664) [29].

In the same operating conditions with the FRAP test, Bouabid and collaborators found that the aqueous macerate of *Atractylis gummifera L* showed the strongest antioxidant activity (102.5 ± 1.66 mg TE/g E) [13]. The macerated acetone extract of *Juglans regia* bark showed the best antioxidant activity (759.11 ± 0.27 *µ*g TE/mg E) [14]. In addition, a phytochemical study on the aerial part of *Ajuga iva* subsp. revealed that the methanolic extract had a reducing power of 22.70 ± 0.19 mg TE/g E [15]. Another phytochemical study conducted on *Anabasis aretioides* of the Chenopodiaceae family showed that the methanolic macerate had the highest antioxidant activity (99.73 ± 3.570 *µ*g TE/mg E) [16].

#### 4.4.5. Reducing Power Assay

Concerning the reducing power (RP) test, we found that the iron reduction profile of the aqueous extracts increases with the increase of temperature; this increase is more marked for the decoctate with a value of 21.89 ± 1.04 Ug E AA/mg E, and this same extract showed a high content of phenolic compounds that are probably responsible for its reducing power. According to El Moussaoui and collaborators, the presence of hydroxylated compounds in the phytochemicals of plant extracts gives them a reducing power and they can be used as electron donors [69].

For the organic extracts, we found that the reducing capacity is proportional to the increase of the polarity of the extracts. The highest reducing power was recorded by the methanolic extract and the methanolic macerate with a statistically nonsignificant difference. In the secondary metabolite assay performed, these two extracts showed higher contents of total polyphenols and flavonoids. The ethyl acetate and chloroform extracts also expressed a high reducing power with a nonsignificant difference; although they had lower quantities of polyphenols, but they had the highest contents of catechic tannins compared to the other organic extracts, which are probably responsible for the reducing power for these two extracts.

A comparison with studies conducted in our laboratory under the same operating conditions on the RP test showed that the aqueous macerated of *Atractylis gummifera L* had the highest antioxidant activity with the PR test (96.15 ± 1.12 mg EAA/g E) [13]. For *Juglans regia*, acetone macerate has the best antioxidant activity (685.68 ± 0.82 *µ*g EAA/g E) [14]. In addition, the methanolic extract of *Ajuga iva* had the highest reducing power (21.55 ± 0.18 *µ*g AAE/mg E) [15]. Another study conducted on a plant of the same family of *Haloxylon scoparium*, *Anabasis aretioides*, showed that the methanolic macerate had the best antioxidant activity (72.176 ± 0.540 *µ*g AAE/mg E) [16].

### 4.5. Principal Component Analysis (PCA)

According to the results obtained from the correlation matrix, the ABTS test is highly positively correlated with the DPPH test (*r*^2^ = 0.9693), which can be explained by the fact that both tests involve the same mechanisms of action, which consist in giving up electrons or hydrogens to eliminate free radicals. The FRAP test is highly positively correlated with the reducing power (RP) test (*r*^2^ = 0.9845) and with the DPPH (*r*^2^ = 0.9424) and ABTS (*r*^2^ = 0.9713) test. The high positive correlation between all the tests probably testifies to the presence in our extracts of antioxidant molecules which can intervene by two types of reaction mechanisms. In the FRAP and RP tests, there is a reduction of Fe(III), based only on electron transfer, whereas in the DPPH and ABTS tests, the radicals can be neutralised either by direct reduction via electron transfer or by radical scavenging via hydrogen atom transfer [70]. Similar results were obtained in our laboratory with other plants from the region of Taza, Morocco, and reported by Senhaji and collaborators showing the presence of a strong correlation among DPPH, ABTS, FRAP, and PR tests realised on *Ajuga iva* and on *Anabasis aretioïdes* which belong to the same family of *Haloxylon scoparium*, Chenopodiaceae [15,16].

The four antioxidant activity tests, DPPH, ABTS, FRAP, and PR, had shown a strong positive correlation with the total polyphenol content of the aqueous and organic extracts; this correlation suggests that these phenolic compounds thus contribute to antioxidant power by two mechanisms. They have redox properties allowing them to act as both hydrogen and electron donating agents [71]. A study by Kourouma and collaborators on twenty-five sweet potato varieties showed a high positive correlation between total phenols and DPPH, ABTS, and FRAP tests [72]. Prior and collaborators also report that the antioxidant capacity assessed by the FRAP test appears to be related to the degree of hydroxylation and conjugation capacity of polyphenols [70]. According to Lv and collaborators, the high antioxidant activities exhibited by plant extracts are due to the presence of polyphenolic compound [73]. Other studies have not established this correlation and have reported that antioxidant activity is positively correlated with the structure of polyphenols [74].

In the same operative conditions, works carried out in our laboratory on other plants of the region of Taza and reported by Boulfia and his collaborators have revealed that phenolic compounds, flavonoids, and tannins are strongly correlated with the antioxidant activity of *Juglans regia* [13]. In addition, Senhaji and collaborators showed a strong correlation among DPPH, ABTS, FRAP, and PR assays carried out on the aerial part of *Ajuga iva* subsp. pseudoiva and on the aerial part of *Anabasis aretioides*, a plant of the Chenopodiaceae family [15,16].

Our results from PCA analysis also show a strong positive correlation between total polyphenol content and flavonoid content, which probably indicates that total polyphenols in the aerial part are predominantly in the form of flavonoids. In concordance with our results, a recent study by Senhaji and her collaborators reported a strong positive correlation between total polyphenol and flavonoid content in the aerial part of *Ajuga iva* [15].

The study of the antihyperglycaemic activity *in vitro* showed a high correlation between the *a*-amylase inhibitory activity and the DPPH (*r*^2^ = 0.8094), ABTS (*r*^2^ = 0.8237), FRAP (*r*^2^ = 0.8115), and PR (*r*^2^ = 0.8508) tests. The correlation between antioxidant activity and antidiabetic activity could be explained, on the one hand, by the particularity of the molecules contained in the aerial part of *Haloxylon scoparium* to have both antioxidant and antidiabetic power and, on the other hand, by the existence of a link between oxidative stress and diabetes. Reactive oxygen species (ROS) can participate in the development of diabetes by altering the action of insulin and destroying the beta cells of the pancreas [75]. A study conducted in Iran on *R. turkestanicum* reported a high correlation between DPPH assay and inhibitory activity by *a*-amylase (*r*^2^ = 0.897) [75].

The *a*-amylase is strongly positively correlated with total polyphenol (*r*^2^ = 0.7721) and flavonoid (*r*^2^ = 0.7162) content. According to Sales et al., polyphenols and flavonoids inhibit the enzyme *a*-amylase through the formation of hydrogen bonds between its hydroxyl groups and the residues of the binding site of this enzyme [76].

The *in vitro* inhibitory activity by the enzymes *a*-glucosidase and *ß*-galactosidase is moderately positively correlated with the H_2_O_2_ antioxidant activity test with values of *r*^2^ = 0.4885 and *r*^2^ = 0.0412, respectively. A study conducted in Malaysia reported the existence of a strong correlation between antioxidant activity and *a*-glucosidase assay of *Ficus deltoidea* water fraction (*R* = 0.998) [77].

According to the results presented in this study, among the organic extracts tested, we found that the methanolic extract with Soxhlet showed high antioxidant and antidiabetic activity compared to the other organic extracts prepared. Similarly, for the aqueous extracts, it was the decoctate that showed high antioxidant and antidiabetic capacity among the other aqueous extracts. It seems from these results that polarity and temperature would play a crucial role in extracting molecules that are responsible for the antioxidant and antidiabetic activity of the aerial part of *Haloxylon scoparium*.

## 5. Conclusion

The results obtained in this study show that the aerial part of *Haloxylon scoparium* is rich in mineral elements (Fe, k, Mg, P, Na, Cu, Ca, and Sr), which may be responsible for the biological effects found in this part of the plant. Furthermore, the phytochemical screening carried out by means of characterisation reactions revealed the richness of the studied aerial part of the *Haloxylon scoparium* plant in secondary metabolites: alkaloids, tannins, saponins, flavonoids, quinones, and anthracenosides.

The quantification by spectrophotometric methods of the contents of secondary metabolites showed that the extracts tested have high contents of total polyphenols, flavonoids, and catechic tannins which may confer biological and pharmacological activities to the plant. This contributes to confirm its use in traditional medicine for the treatment of several anomalies.

The *in vitro* evaluation of the antidiabetic activity showed that the decoctate has a higher inhibitory capacity on *a*-glucosidase than acarbose, ethyl acetate extract has the best inhibitory capacity on *ß*-galactosidase and *a*-amylase, and methanolic extract and macerated methanol had an inhibitory effect on *a*-glucosidase.

The study of antioxidant properties of aqueous and organic extracts showed that the aerial part of *Haloxylon scoparium* has free radical scavenging potential. The decoctate showed the best antioxidant activity among the aqueous extracts and for the organic extracts, the methanolic extract and the macerated methanol showed the highest antioxidant activity, respectively.

The principal component analysis (PCA) showed a positive correlation of the antidiabetic activity with the polyphenol and catechic tannin content and with the antioxidant activity tests. PCA also showed a high positive correlation between the four antioxidant activity tests, DPPH, ABTS, FRAP, and PR, performed on the aerial part of *Haloxylon scoparium* and between the antioxidant power and the content of total polyphenols and flavonoids.

These results represent a first step in the research on the mineral composition and active principles of the secondary metabolites and their antioxidant activity of *Haloxylon scoparium* and constitute a support to carry out, on the one hand, *in vivo* tests to confirm the results obtained *in vitro* and, on the other hand, to continue the chemical study in order to identify precisely the compounds responsible for the biological and pharmacological activities of the plant.

## Figures and Tables

**Figure 1:** *Haloxylon scoparium* (pictures taken on 17 July 2019 in Taddart located 42.1 km from the city of Taza; geographical coordinates: N 34°12.530′, W 003°32.917′).

**Figure 2:** Correlation circle of the variables and the positioning of the individuals on the first main plane (83.39% information) (D: decocted; I: infused; MA: aqueous macerated; MM: methanolic macerated; M: methanolic extract; AE: ethyl acetate extract; CH: chloroformic extract; EP: petroleum ether extract; G1: Group 1; G2: Group 2; G3: Group 3; DPPH: 2,2-diphenyl-1-picrylhydrazyl; H_2_O_2_: hydrogen peroxide; ABTS: 2,2′-azino-bis(3-ethylbenzothiazoline-6-sulphonic acid); FRAP: iron reducing antioxidant power; PR: iron reducing power; TP: total polyphenols; TF: total flavonoids; TCT: total catechic tannins).

**Table 1:** Mineral composition of the aerial part of *Haloxylon scoparium.*

Mineral elements	Fe	K	Mg	P	Na	Cu	Ca	Sr	Se	Zn
Content in mg/kg of dry matter	**60909.00**	**27452.10**	**10059.90**	**1125.39**	**1054.65**	438.93	313.29	280.23	3.00	3.00

Fe: iron; K: potassium; Mg: magnesium; P: phosphorus; Na: sodium; Cu: copper; Ca: calcium; Sr: strontium; Se: selenium; Zn: zinc.

**Table 2:** Yields of aqueous and organic extractions of the aerial part of *Haloxylon scoparium*.

	Extracts	Yield in %
Aqueous extracts	**Decocted**	**16**
	Infused	8
	Macerated	5

Organic extracts	**Methanol extract**	**14.35**
	**Macerated methanol**	**10.68**
	Ethyl acetate extract	2.17
	Chloroform extract	2.34
	Petroleum ether extract	0.89

**Table 3:** Phytochemical screening of the powder and the aqueous and organic extracts of the aerial part of *Haloxylon scoparium*.

Plant powder and aqueous and organic extracts		Catechic tannins	Gallic tannins	Flavonoids	Saponins	Alkaloids	Sterols	Anthracenosides	Anthraquinones	Free quinones
Powder of the aerial part of the plant		+++	−	++	++	+++	−	+	−	+

Aqueous extracts	Decocted	**+++**	−	**++**	**+++**	**+++**	−	−	−	−
	Infused	**+++**	−	**++**	**+++**	**+++**	−	−	−	−
	Macerated	**+++**	−	**++**	**++**	**+++**	−	−	−	−

Organic extracts	Methanol	**++**	−	**++**	**++**	**+++**	−	**++**	−	**++**
	Macerated methanol	**++**	−	**++**	**++**	**+++**	−	**++**	−	**++**
	Ethyl acetate	**++**	−	−	−	**+++**	−	−	−	**+**
	Chloroform	**++**	−	−	−	**+++**	−	−	−	**+**
	Petroleum ether	**++**	−	−	−	**+++**	−	−	−	−

**+++**: very abundant; **++**: moderately abundant; **+**: present; **−**: absent.

**Table 4:** Contents of total polyphenols, flavonoids, and catechic tannins in aqueous and organic extracts of the aerial part of *Haloxylon scoparium*.

Extracts		Total phenolic content (*µ*g GAE mg^−1^E)	Total flavonoid content (*µ*g QE mg^−1^E)	Total catechic tannin content (*µ*g CE mg^−1^E)
Aqueous	Decocted	**6.83** **±** **0.04**^***a***^	**306.59** **±** **4.35**^***a***^	**3.78** **±** **0.35**^***a*,*b*,*c*,*e***^
	Infused	3.81 ± 0.21^*a*,*b*^	228.67 ± 10.87^*b*^	1.1 ± 0.13^***a*,*c***^
	Macerated	3.96 ± 0.07^*a*,*b*^	135.78 ± 3.57^*c*^	2.25 ± 0.12^***a*,*b*,*c***^

Organic	Methanol	**161.65** **±** **1.52**^***c***^	**612.47** **±** **10.10**^***d***^	6.02 ± 0.11^*b*^
	Macerated methanol	147.11 ± 6.11^***d***^	**641.03** **±** **7.8**^***d***^	0.26 ± 0.2^*c*^
	Ethyl acetate	54.24 ± 2.70^*e*^	416.73 ± 10.18^*e*^	**23.69** **±** **0.6**^***d***^
	Chloroform	49.42 ± 1.02^*e*^	263.25 ± 2.59^*b*^	21.25 ± 2.25^*d*^
	Petroleum ether	11.30 ± 1.58^*b*,*f*^	168.3 ± 7.91^*c*^	7.55 ± 1.18^*b*,*e*^

All results expressed are mean of three individual replicates (*n* = 3 ± SEM). Values with the same letter superscript in the same row are not significantly different (*p* < 0.05).

**Table 5:** IC50 (µg/mL) of *a*-amylase, *a*-glucosidase, and *ß*-galactosidase inhibitory activity of aqueous and organic extracts of the aerial part of *Haloxylon scoparium.*

Extracts	*α*-Amylase	*α*-Glucosidase	*β*-Galactosidase
Decocted	**66855.66** **±** 10.51^a,b,c^	**181.7** **±** **21.15**^**a**^	1361.66 ± 188.40^a,b,c^
Infused	78892.33 ± 14.44^a,b,c^	225.44 ± 58.43^a,b^	**915.23** **±** **68.86**^a^
Macerated	80277.33 ± 7.61^a,b^	202.10 ± 75.44^a,b^	1072.73 ± 369.28^a,c^
Methanol	56156.33 ± 2.58^b,c^	**193.4** **±** **8.57**^a,b^	**1735.66** **±** **269.50**^a,b^
Macerated methanol	**46351** **±** 4.88^b,c^	200.86 ± 1.99^a,b^	1984.66 ± 61.65^a,b^
Ethyl acetate	39096.66 ± 4.17^b,c^	235.9 ± 35.56^a,b^	1601.66 ± 107.21^a,b^
Chloroform	51261 ± 4.78^b,c^	341.73 ± 13.92^a,b^	**1707.66** **±** **12.99**^a,b^
Petroleum ether	66601 ± 12.21^b,c^	357.16 ± 2.50^a,b^	1819.66 ± 172.29^a,b,c^
Acarbose	616.33 ± 5.00^d^	195 ± 6.12^a,b^	—
Quercetin	—	—	171.16 ± 5.00^d^

All results expressed are mean of three individual replicates (*n* = 3 ± SEM). Values with the same letter superscript in the same row are not significantly different (*p* < 0.05).

**Table 6:** Results of *in vitro* antioxidant activity of aqueous and organic extracts of the aerial part of *Haloxylon scoparium* via five tests: H_2_O_2_, DPPH, ABTS, FRAP, and PR.

Extracts		H_2_O_2_ (%)	DPPH (IC50)	ABTS (ug E AA/mg E)	FRAP (ug E T/mg E)	PR (ug E AA/mg E)
Aqueous extracts	Decocted	**16.21** **±** **0.39**^*a*^	**439.3** **±** **7.74**^***a***^	**8.20** **±** **0.01**^*a*^	**37.66** **±** **1.29**^*a*,g^	**21.89** **±** **1.04**^*a*^
	Infused	8.78 ± 0.41^*b*^.^*e*^	518.96 ± 5.66^*b*^	5.14 ± 0.37^*a*,*d*^	27.94 ± 1.08^*a*,*b*,g^	14.09 ± 0.74^*a*^
	Macerated	4.15 ± 0.43^*c*^	582.8 ± 14.72^*c*^	3.99 ± 0.26^*a*,*d*^	17.81 ± 3.50^*b*,g^	6.63 ± 0.40^*a*^

Organic extracts	Methanol	**20.91** **±** **0.27**^***d***^	**39.63** **±** **2.03**^***d***^	**50.75** **±** **0.72**^***b***^	**163.37** **±** **1.52**^*c*^	**116.18** **±** **8.19**^*b*^
	Macerated methanol	7.36 ± 0.09^*e*^	57.87 ± 1.50^*d*,*e*^	47.71 ± 1.21^***b***^	124.08 ± 6.97^*d*^	110.11 ± 7.47^*b*^
	Ethyl acetate	7.26 ± 0.11^*e*^	62.27 ± 1.82^*d*,*e*^	39.74 ± 1.41^***c***^	106.14 ± 5.26^*e*^	79.27 ± 4.78^*c*^
	Chloroform	5.84 ± 0.39^*e*,*f*^	72.00 ± 1.88^***e***^	36.99 ± 1.34^***c***^	85.02 ± 2.96^*f*^	59.35 ± 0.65^*c*^
	Petroleum ether	5.76 ± 0.4^*e*,*f*,*c*^	297.8 ± 1.15^***f***^	1.72 ± 0.53^***d***^	24.51 ± 0.53^g^	0.96 ± 0.3^*a*^

Reference standards	Ascorbic acid	**14.35** **±** **0.002**^g^	**0.17** **±** **0.02**^**g**^	—	—	—
	BHT		**1.59** **±** **0.13**^**g**^			
	Trolox		**1.75** **±** **0.09**^**g**^			

All results expressed are mean of three individual replicates (*n* = 3 ± SEM). Values with the same letter superscript in the same row are not significantly different (*p* < 0.05).

**Table 7:** Correlation coefficient between the antioxidant variables, *a*-amylase, *a*-glucosidase, and *ß*-galactosidase enzyme inhibitory activities, and the chemical contents of aqueous and organic extracts of the aerial part of *Haloxylon scoparium*.

Variables	H_2_O_2_	DPPH	ABTS	FRAP	RP	Total phenolics	Flavonoids	Catechic tannins	*α*-Amylase	*α*-Glucosidase	*β*-Galactosidase
H_2_O_2_	**1**										
DPPH	0.2581	**1**									
ABTS	0.3023	**0.9693**	**1**								
FRAP	0.4676	**0.9424**	**0.9713**	**1**							
RP	0.3906	**0.9255**	**0.9809**	**0.9845**	**1**						
Total phenolics	0.4477	**0.8563**	**0.8944**	**0.9372**	**0.9429**	**1**					
Flavonoids	0.5243	**0.8055**	**0.8567**	**0.8730**	**0.8983**	**0.9416**	**1**				
Catechic tannins	−0.2149	0.4813	0.3640	0.2451	0.1921	−0.0338	−0.0433	**1**			
*α*-Amylase	0.1604	**0.8094**	**0.8237**	**0.8115**	**0.8508**	**0.7721**	**0.7162**	0.1979	**1**		
*α*-Glucosidase	0.4885	−0.0822	0.1413	0.2234	0.2832	0.2696	0.2851	−0.5792	0.1484	**1**	
*β*-Galactosidase	0.0412	−0.6996	−0.5983	−0.5705	−0.5658	−0.6320	−0.5357	−0.2659	−0.7078	0.2847	**1**

## Data Availability

The experimental data used to support the findings of this study are incorporated into the article.

## Abbreviations

*H. scoparium*: *Haloxylon scoparium*
ROS: Reactive oxygen species
H_2_O_2_: Hydrogen peroxide scavenging assay
TEAC or ABTS: Trolox equivalent antioxidant capacity method/ABTS radical cation decolorization assay
FRAP: Ferric reducing antioxidant power assay
RP: Reducing power method
DPPH: 1,1-diphenyl-2-picrylhydrazyl scavenging activity
PCA: Principal component analysis
ANOVA: Analysis of variance
IC50: Concentration that causes 50% inhibition.
